The article "Can the genes communicate with each other after birth? An international cross‐sectional study" was published in 2023. Journal: Health Sci Rep.

# Can the genes communicate with each other after birth? An international cross‐sectional study

**DOI:** 10.1002/hsr2.1084

**Published:** 2023-01-30

**Authors:** Hashim Talib Hashim, Ali Talib Hashim, Abubakar Nazir, Usama Afzaal, Awais Nazir, Ahmed Dheyaa Al‐Obaidi

**Affiliations:** ^1^ College of Medicine University of Baghdad Baghdad Iraq; ^2^ Department of Medicine Golestan University for Medical Sciences Gorgan Iran; ^3^ Department of Medicine King Edward Medical University Lahore Pakistan

**Keywords:** DNA, genes, genes' communication, genes' waves, genetics, genomic

## Abstract

**Background:**

Various factors contribute to the pathogenesis of a disease. These include genetic factors, family history, and some idiopathic causes. Genetic makeup has an important role in the progression of disease. This is due to mutations in genetic material, that is, deoxyribonucleic acid (DNA).

**Methodology:**

This is a cross‐sectional study that involved 5000 participants distributed across 250 countries. All the participants were randomly selected and asked to fill out the online survey. All the participants were fully informed about the study's purpose before providing their consent.

**Results:**

The participants were distributed among 250 countries. Their age mean (standard deviation) is 46.7 (12.4). We discovered a significant difference between those who have genetic or congenital diseases and those who have a family history of the disease. Also, there is a statistically significant difference between the recurrence of the disease and the duration of the visits of close relatives who have the same disease.

**Conclusion:**

The study suggests that there might be some ways, through gene waves or the environment, in which a gene changes the expression of other genes of similar sequence in different individuals when the required period of contact is provided. In the future, this theory might explain the idiopathic nature of some diseases.

## 1 INTRODUCTION

Various factors contribute to the pathogenesis of a disease. These include genetic factors, family history, and some idiopathic causes. Genetic makeup has an important role in the progression of disease. This is due to mutations in genetic material, that is, deoxyribonucleic acid (DNA). Differences in DNA can make an individual more susceptible to some diseases for example, a certain type of cancer.^1^ On the other hand, these changes could make a person less susceptible to some disorders, like diabetes. The role of various environmental factors, like lifestyle, is significant in many diseases, like the role of diet and exercise in diabetic patients. However, the body's response to environmental factors varies depending on its genetic constitution.^1^ The immune system is greatly influenced by genetic factors. These factors cause variation in each individual's immune system, which in turn determines the individual's immunity against pathogens.^1^, ^2^ The majority of cancers are caused by genetic mutations and changes. These mutations are affected by genetic and environmental factors. Among various possible factors causing disease in humans, family history is one of the most important factors leading to common disease complexes like cancer, heart disease, psychiatric illnesses, diabetes, and autoimmune disorders.^2^ A person's risk of developing a disease can be predicted by family history. Genetic variation inherited by the individual can lead to the pathogenesis of disease.^2^ A complete understanding of the genome and genetics is vital for evaluating the progression of disease and devising a therapeutic strategy for prevention. interaction between environmental initiating factors and genetic factors is also involved in disease progression.^3^ Some diseases have a seasonal onset, like allergies caused by environmental factors. Exposure to ultraviolet light can cause skin disorders in susceptible individuals.^3^ Risk for environmental diseases is increased by interactions among genetic factors, acquired susceptibility, and environmental factors.

The article "Can the genes communicate with each other after birth? An international cross‐sectional study" was published in 2023. Journal: Health Sci Rep.

## 2 METHODOLOGY

### 2.1 Study design

We have undertaken a cross‐sectional, international, multicenter study, using an online self‐administered questionnaire, on the cohort composed of participants who were randomly chosen from 250 countries.

### 2.2 Setting

The survey was conducted in each country had a center, and there was an administrator for each country to select the cases.

### 2.3 Participants

An online survey was conducted randomly among the general population and included only those who completed the survey properly. There was a consent form for participants at the beginning of each survey and an explanation of the study. Ethical approval was obtained from the ethical committee of the University of Baghdad, College of Medicine.

### 2.4 Variables

The questionnaire consisted of 30 questions divided into two sections. The answers were divided into single answers and multiple‐choice answers for both quantitative questions and qualitative questions.

### 2.5 Study size

The study involved 5000 participants distributed in 250 countries.

### 2.6 Statistical method

We used SPSS version 24 in finding a relationship between our variables for significance and correlation. In the analysis, the *χ* ^2^ and Fisher's tests were used.

## 3 RESULTS

The participants were 5000 distributed among 250 countries. Their age mean (standard deviation) is 46.7 (12.4). Table 1 demonstrates the demographic data related to the participants.

The article "Can the genes communicate with each other after birth? An international cross‐sectional study" was published in 2023. Journal: Health Sci Rep.

**Table 1:** The demographic data of the participants.

Age group	
<30 years	70% (*n* = 3500)
30–60 years	24% (*n* = 1200)
>60 years	6% (*n* = 300)
Gender	
Male	41.56% (*n* = 2078)
Female	40.2% (*n* = 2010)
Others	18.24% (*n* = 912)
Educational level completed	
Illiterate	24.44% (*n* = 1222)
Primary school	20.02% (*n* = 1001)
High school	42.38% (*n* = 2119)
College or more	13.16% (*n* = 658)
Monthly income	
<1000$	77.74% (*n* = 3887)
1000–5000$	20.26% (*n* = 1013)
>5000$	2% (*n* = 100)
Religion	
Christians	43.12% (*n* = 2156)
Muslims	23.34% (*n* = 1167)
Hinduism	14.04% (*n* = 702)
Jewish	10.06% (*n* = 503)
No religion	1.44% (*n* = 72)
Others	8% (*n* = 400)
Race	
White	48.34% (*n* = 2417)
American African	12.18% (*n* = 609)
Asian	17.8% (*n* = 890)
Arabic	18.28% (*n* = 914)
Black	2.1% (*n* = 105)
Others	1.3% (*n* = 65)
Marital status	
Married	72.9% (*n* = 3645)
Unmarried	27.1% (*n* = 1355)
Number of children	
<3 children	59.26% (*n* = 2963)
3–5 children	24.88% (*n* = 1244)
>5 children	15.86% (*n* = 793)
Chronic illnesses	
Diabetes melletus	69.72% (*n* = 3486)
Hypertension	79.64% (*n* = 3982)
Cancer	47.08% (*n* = 2354)
Handicap	20.04% (*n* = 1002)
Epilepsy	10.16% (*n* = 508)
Heart diseases	55.88% (*n* = 2794)
Renal diseases	38.14% (*n* = 1907)
Liver diseases	21.34% (*n* = 1067)
Others	40.88% (*n* = 2044)
Living status	
With family (parents and brothers)	47.38% (*n* = 2369)
Independent	39.64% (*n* = 1982)
Homeless	12.98% (*n* = 649)

The questionnaire involved 16 questions about the role of genes in the disease's transmission and the cofounders; Table 2 demonstrated the percentages of the responses for each question.

**Table 2:** The questions.

Q1: Do have any genetic disease?	
Yes	73.08% (*n* = 3654)
No	26.92% (*n* = 1346)
Q2: Do you have any congenital disease?	
Yes	26.52% (*n* = 1326)
No	73.48% (*n* = 3674)
Q3: Does one of the diseases above exist in your family (first degree or second degree)?	
Yes	79.56% (*n* = 3978)
No	20.44% (*n* = 1022)
Q4: Do you live in the same city or country of your family?	
The same city	53.08% (*n* = 2654)
The same country	46.92% (*n* = 2346)
Q5: Do you share any of your diseases with your brothers, sisters, parents?	
Yes	32.74% (*n* = 1637)
No	67.26% (*n* = 3363)
Q6: How many times do you visit your family?	
Weekly	40% (*n* = 2000)
Monthly	40.66% (*n* = 2033)
Yearly	19.34% (*n* = 967)
Q7: For how long do you stay close to them?	
For days	60.32% (*n* = 3016)
Weeks	20.24% (*n* = 1012)
Months	10.74% (*n* = 537)
Years	8.7% (*n* = 435)
Q8: How many times do your brothers or sister visit your family?	
Weekly	63.86% (*n* = 3193)
Monthly	20.46% (*n* = 1023)
Yearly	15.68% (*n* = 784)
Q9: For how long do they stay close to them?	
Days	15.88% (*n* = 794)
Weeks	34.9% (*n* = 1745)
Months	47.1% (*n* = 2355)
Years	2.12% (*n* = 106)
Q10: Have you been treated from the disease?	
Yes	42.98% (*n* = 2149)
No	57.02% (*n* = 2851)
Q11: If yes, have the disease recurred to you?	
Yes	69.56% (*n* = 3478)
No	30.44% (*n* = 1522)
Q12: If yes, when the disease recurred, were you living with your family?	
Yes	83.56% (*n* = 4178)
No	16.44% (*n* = 822)
Q13: Does the diseased person from your family treated?	
Yes	57.42% (*n* = 2871)
No	42.58% (*n* = 2129)
Q14: Does the disease recur to him or her?	
Yes	62.06% (*n* = 3103)
No	37.94% (*n* = 1897)
Q15: After how much time, it recurs to you?	
After months	10% (*n* = 500)
After years	30% (*n* = 1500
Never recur	39.86% (*n* = 1993)
I am not sure	20.14% (*n* = 1007)
Q16: After how much time, it recurs to the person from your family?	
After months	34.12% (*n* = 1706)
After years	43.18% (*n* = 2159)
Never recur	9.26% (*n* = 463)
I am not sure	13.44% (*n* = 672)

In Figure 1, we can see the relationships between the duration of staying close to the parents or close relatives and the duration of the diseases and their recurrence.

The article "Can the genes communicate with each other after birth? An international cross‐sectional study" was published in 2023. Journal: Health Sci Rep.

**Figure 1:** The relationship between the duration of staying with families and the time of recurrence after treatment. We see that all the durations have caused the recurrence to be increased except for the days for which no relationship exists.

We found a significant difference between those who have genetic diseases or congenital diseases and the incidence of the disease in their families (Table 3). Also, there is a statistically significant difference between the recurrence of the disease and the duration of the visits of close relatives who have the same disease.

**Table 3:** The *p*‐value of *χ* ^2^ testing results between variables.

The first variable	The second variable	*p* Value
Q3	Q1, Q2	0.01, 0.00
Q11	Q6, Q7	0.0, 0.03
Q14	Q6	0.02
Q15	Q7	0.00
Q16	Q9	0.04
Q11	Living status	0.01

## 4 DISCUSSION

Our study seeks to discover the relationship between the period of stay with the family having or not having genetic disease and the recurrence of disease after appropriate management in an international population sample to determine whether genes communicate with each other after birth between individuals. This study only emphasizes the degree of association between the length of stay with families and disease recurrence and has nothing to do with a causal relationship. We recruited a large sample of individuals of varying ages with a history of genetic disease in them or family members living away from the family and found that whether visiting and staying close to your family members has an impact on disease behavior and how long disease recurs in subjects. There is a significant association between the individual having a congenital or genetic disease and the family history of disease. First‐ and second‐degree relatives can be found in a family tree. Structural and functional abnormalities that happen during intrauterine life result in congenital disease. It can appear during the perinatal period or later in life. Genetic diseases are under the umbrella of congenital diseases.^4^ We discovered a strong association between disease recurrence and visiting family frequently when we compared individuals with genetic disease in remission who visit their family and spend time with them closely to those who do these things less frequently in their lives. There is also a strong link between disease recurrence and spending time with family. It implies that visiting your family more frequently and spending more time with them may increase your chances of disease recurrence. This suggests that genes most likely communicate with each other after birth. Reciprocally, a person may have siblings with some sort of genetic disease living together with their family, and his visit may impact the behavior of the disease. This study provides strong evidence that increasing the number of visits to the family increases the chances of recurrence in their siblings. In fact, this is another clue that genes may communicate with each other after birth. This suggests that when an environment is changed to one in which factors are present, this may influence the expression of genes and thus the phenotype. In this study, for example, we have disease recurrence as a dependent variable and period of contact with family as an independent parameter. An individual with genetic disease most likely has a family history (*p* value between 0.01 and 0.00), which means that there are higher chances that such genes are present in their family. These genes, controlling the internal environment as well as the external environment through their expression, might have created such an environment that when an individual with disease has a long period of contact with their family members, their genetic expression is modified and disease recurs in them, considering only the genes having similar sequences.^2^ Thus, there is a hypothesis that genes from blood relatives may influence the expression of one's genes and thus the recurrence of disease.

The article "Can the genes communicate with each other after birth? An international cross‐sectional study" was published in 2023. Journal: Health Sci Rep.

Duration of time is also very important for both the period of contact and the time after a disease recurs. Our study also has strong evidence for this argument. Individual disease incidence increases with the length of stay with family. This is particularly important when an individual has a period of contact stretching over weeks, months, or years. When the period of contact is encompassed over several days, it doesn't have a significant effect. It means that there is no significant relationship between disease recurrence and period of contact when stay is limited to a few days. It may be due to the fact that genes require a considerable amount of time for their expression or that their expression is influenced by environmental factors. A specific time is required for genetic expression. It is different for different genes. So, genes require a certain amount of time to influence their effect on other genes, and these genes require a certain amount of time to alter their expression.^5^ Thus, we can assume that days are not enough for genes to have an influence on other genes. This requires a specific amount of time. Genes can communicate with each other after birth only if the period of contact is stretched over the required period of time, and our study has evidence to support this argument. Our study also finds a strong link between living status and disease recurrence (*p* value of 0.01). Studies suggest that persons with improved living status and social support have been shown to have a better outcome, decreased mortality, and an increased disease‐free interval.^6^ Also, the quality of life is enhanced. Because the environment has a large influence on disease behavior, your living situation may have influenced the disease's recurrence. We simply wanted to find a relationship between genes with similar sequences and each other in different individuals by considering family history of inherited diseases in this study. we have listed some evidence that supports our hypothesis. We think that there may be some types of communication signals—we called them “gene waves”—through which genes communicate with each other. We have considered the distance of separation, the period of contact, and the duration after which recurrence occurs. The study suggests that there might be some ways, through gene waves or the environment, in which a gene changes the expression of other genes of similar sequence in different individuals when the required period of contact is provided. In the future, this theory might explain the idiopathic nature of some diseases. Of course, our study has some limitations as well. We tried our best to control the confounding by matching the variables as far as we could, but there may be some variables that might have influenced the results that should be discovered by further research. As our study is novel in nature, there is very little literature available on this, and a lot of debate is required to find out whether there is real communication or not. As our study is cross‐sectional in nature, we have only found the associations between the variables, not the casual relationships between them.

The article "Can the genes communicate with each other after birth? An international cross‐sectional study" was published in 2023. Journal: Health Sci Rep.

## 5 CONCLUSION

We simply wanted to find a relationship between genes with similar sequences and each other in different individuals by considering family history of inherited diseases in this study. We have listed some evidence that supports our hypothesis. We think that there may be some types of communication signals—we called them “gene waves”—through which genes communicate with each other. We have considered the distance of separation, the period of contact, and the duration after which recurrence occurs. The study suggests that there might be some ways, through gene waves or the environment, in which a gene changes the expression of other genes of similar sequence in different individuals when the required period of contact is provided. In the future, this theory might explain the idiopathic nature of some diseases.

## AUTHOR CONTRIBUTIONS

**Hashim Talib Hashim**: Conceptualization; data curation; formal analysis; methodology; project administration; resources; supervision; validation; visualization; writing – review and editing. **Ali Talib Hashim**: Conceptualization; methodology; writing – original draft. **Abubakar Nazir**: Formal analysis; software; writing – original draft. **Usama Afzaal**: Data curation; software; writing – original draft. **Awais Nazir**: Data curation; software; writing – original draft. **Ahmed Dheyaa Al‐Obaidi**: Formal analysis; methodology; validation; writing – review and editing.

## CONFLICT OF INTEREST STATEMENT

The authors declare no conflict of interest.

## ETHICS STATEMENT

Ethical approval was obtained from the ethical committee in the University of Baghdad, College of Medicine. Patients' consents were given before recruitment.

## TRANSPARENCY STATEMENT

The lead author Hashim Talib Hashim affirms that this manuscript is an honest, accurate, and transparent account of the study being reported; that no important aspects of the study have been omitted; and that any discrepancies from the study as planned (and, if relevant, registered) have been explained.

## Data Availability

Data will be available upon reasonable request.
